# Logic Design and Power Optimization of Floating-Point Multipliers

**DOI:** 10.1155/2022/6949846

**Published:** 2022-01-07

**Authors:** Na Bai, Hang Li, Jiming Lv, Shuai Yang, Yaohua Xu

**Affiliations:** Key Laboratory of Computational Intelligence and Signal Processing, Ministry of Education (Anhui University), School of Integrated Circuit, Anhui University, School of Electronic Information Engineering, Anhui University, Hefei 230601, China

## Abstract

Under IEEE-754 standard, for the current situation of excessive time and power consumption of multiplication operations in single-precision floating-point operations, the expanded boothwallace algorithm is used, and the partial product caused by booth coding is rounded and predicted with the symbolic expansion idea, and the partial product caused by single-precision floating-point multiplication and the accumulation of partial products are optimized, and the flowing water is used to improve the throughput. Based on this, a series of verification and synthesis simulations are performed using the SMIC-7 nm standard cell process. It is verified that the new single-precision floating-point multiplier can achieve a smaller power share compared to the conventional single-precision floating-point multiplier.

## 1. Introduction

According to a study by Stanford University, the demand for arithmetic power in artificial intelligence has doubled every three to four months since 2012, a rate that has surpassed Moore's law (doubling the number of transistors in a chip every 18 months) [1]. That is, the current rate of Moore's law has lagged far behind the speed of the growth in demand for computing power, relying solely on the progress of process technology that has been entirely unable to meet the demand for computing power growth. According to Intel's latest study, for computationally intensive applications, floating-point operations account for 75% of processor core power consumption and 45% of total processor power consumption [2], as shown in Figure 1, while its operator power consumption accounts for 39.57% in Think-II, an artificial intelligence inference chip developed by the first team of the Institute of Microelectronics at Tsinghua University [3]. From this, it can be seen that floating-point operation is a module with a very large power consumption ratio in big data computing, so it is significant to reduce the power consumption of floating-point operation.

As an important indicator of scientific computing capability, floating-point arithmetic is an important computing method for processing various information in today's electronic information tools. Floating-point numbers have a large dynamic range compared to fixed-point numbers; however, the structure is more complex and power consumption is higher, so it is a meaningful breakthrough to achieve multiplicative power optimization of floating-point numbers. In the past, 60% of the performance improvement of microprocessors depended on process advancement [4]; now, we need a breakthrough in design to achieve the demand of arithmetic power growth.

This paper focuses on the power optimization of single-precision floating-point multiplication operations in floating-point operations. The single-precision floating-point multiplication calculation can be divided into three parts, namely, the judgment of symbolic bits, the summation of exponential bits, and the multiplication of trailing bits. The first two conventional designs are similar in this paper, but the core of the design optimization is in the multiplication of trailing bits.

The conventional design for the trailing part of the multiplier is mainly a Wallace tree structure with a combined CSA and 4-2 compressor, mainly in the form of a booth code. Finally, the final product is obtained with an overrunning adder [5].  Figure 2 shows the conventional tail partial multiplier design.

In this paper, we hope to improve the coherent design to reduce the power consumption of single-precision floating-point multipliers.

## 2. Materials and Methods

### 2.1. Ideas and Advantages of the Design Algorithm Based on Boothwallace Tree

For the current design of single-precision floating-point multiplication, this paper divides the design into three parts as the direction of optimization: how to appropriately increase the throughput of data processing when emitting signals; how to process the partial products caused by the multiplication of trailing bits and reduce the number of operations and storage at the same time; and how to effectively reduce the workload of summing and reduce the hyperactive operations in the process of partial product summing.

This design is considered for processing a huge amount of multiplication data operations at 2 GHZ frequency. If we just follow the timing sequence to process one data and then continue to process the next data, such a way is actually very inefficient. Therefore, this paper adopts the form of flowing water to improve the throughput of data processing and increase the frequency of the clock. Although the primary delay (*n∗*(*T*1 + *T*2)) is added in the first stage of processing, the pipelined operation can substantially improve the overall data processing efficiency because the register delay must be smaller than the combinational logic delay. The difference time between the register delay and the combinational logic delay can be saved almost every time the pipelined data processing is done under the huge data processing. The disadvantage of pipelining is that it increases power consumption, area, and hardware complexity. Therefore, while using pipelining to improve data processing efficiency, it is important to weigh the loss of power consumption, area, and software complexity.

The encoding operation of the partial product caused by the trailing bits in the multiplication stage can significantly affect the final power consumption and area. If the partial product is used directly or a simple booth-2 coding operation is done, the power consumption loss and the area occupied are too large. Adopting the booth-4 encoding form can reduce half of the partial product caused by booth-2, compared to the direct use of the partial product form that reduces the part beyond 1/2, which can significantly reduce the time consumption caused by the subsequent operation of partial product, but also can significantly reduce power consumption. Although in the case of booth-4 coding operation, there will be some assignment and logic operations, which will lead to this coding operation will consume a certain amount of time and power consumption, as well as occupy part of the area, still, for a large number of data operations, the increased consumption of this part is much smaller than the consumption saved by the subsequent partial product operation of the data, so this paper uses the booth-4. The symbolic bit expansion method is used in this paper [6]. The symbolic bit expansion can predict the partial product sum form, which can appropriately compress some redundant operations of the partial product sum, and use a certain logical relationship between the two summed partial products to establish the variable relationship, which can compress the area and reduce the power consumption to a certain extent to achieve a comprehensive multiplication of multiple bits, and a large number of partial sums can save a lot of areas and power consumption effect and for subsequent operations can reduce more add operations [7].

In the partial product summation stage, using the direct array summation form or the rounding reservation form will result in a large blanking hypervalue, which will not only occupy a large area but also increase the nonessential addition operations leading to increased power consumption and time. Using the Wallace tree in the form of overlay summation in the form of tree depth reduction will greatly reduce the number of nonessential addition operations and reduce the amount of white space, resulting in a significant improvement in time. Although multiple uses of the full adder can cause a slight loss of power consumption, but for a large amount of data processing, it brings better rate gain and is therefore chosen [8].

### 2.2. Implementation Platform and Implementation Algorithm

#### 2.2.1. Implementation Platform and Process

Figure 3 shows the experimental platform and the validation process [9].

The first step is to build a golden model database in the MATLAB platform about single-precision floating-point multipliers and multiplied numbers and generating control group products. Since the range of single-precision floating-point designs is too wide to be verified by the exhaustive method based on hardware limitations, it is the idea of the design to create a database of golden models as the basis for verification calls. The simple steps are to use the rand function and the num2hex function to generate random data and convert single-precision floating-point data. A database of 100 million multipliers and multiplied numbers are created, saved as num and hex types, respectively, and multiplied together in MATLAB to form a product database as a control group for later testing processes as an accuracy standard. After generating the data, the hist function is used to demonstrate the uniformity of the generated database to ensure that the generated database is the golden model database and reduce the uncontrollable experimental error. The following are the functions for generating random data and converting type functions:

(1) $$\begin{array}{c} a\left(i\right)=f+2*e*\text{rand}\left(1,1,\text{single}\right),\\ a\_\text{temp}=\text{num}2\text{hex}\left(a\left(i\right)\right). \end{array}$$

Under the foundation of the golden model database with good calls, a suitable testbench environment needs to be established as a way to verify the authenticity of the source code logic and debug the source code logic optimization. The platform for design implementation is the NC-Verilog platform. Here, in addition to calling the golden model database and generating the verification product library, the direct window output under the waveform file is also done. The display function is called with embedded precision verification judgments to simplify verification access.

In order to subsequently implement the power consumption parameter analysis and obtain the simulation data for each of the source codes, a synthesizable implementation of the source code is required. The design is implemented in the Design Compiler platform. The original description of the source code is modified, and the source code is reshaped in the specified hardware description language. After invoking the synthesis environment, the synthesis simulation of the source code is realized, and the simulation data of each source code can be obtained, and the required slack data and area data can be extracted as the final control index. In the process of synthesis, the required netlist file is generated as a sample for subsequent calls. It should be noted that the DC environment CLK needs to be annotated when calling Design Ware samples, and the source code constraint in this paper is 2 GHz. Here, this paper relies on the final code to generate the circuit netlist to observe the structure of the circuit diagram.

After generating the required circuit netlist file samples, call the samples to verify them in the testbench environment, noting that it may be necessary to create a process library for import. After verification, the VCD waveform file sample is exported, and the circuit netlist sample and VCD waveform file sample are imported into the PTPX platform to create the required PTPX environment to generate the corresponding power analysis report sample. Based on the samples and the required theory, the source code is designed and optimized, and the optimized samples are saved. And save the Design Ware samples as a control group to achieve the desired results.

#### 2.2.2. Logic Design and Optimization

The basic single-precision floating-point multiplier is built on the basis of the binary floating-point representation formula, which extracts the sign bits, the tail f, and the step code e from the 32-bit binary data, respectively.  Figure 4 represents the arithmetic structure of this 32-bit single-precision floating-point number. The core part is the fixed-point multiplication of the trailing part af:{1′b1, a[22:0]}, bf:{1′b1, b[22:0]}. In the based code, this multiplication structure is the simplest shift judgment flow structure. In the optimization structure, the main thing is also the fixed-point multiplication in the tail part and the optimization of the accuracy in the combination of the final product c parts [10].

The booth-4 encoding has been introduced above to effectively reduce the number of partial products caused by the fixed-point multiplier. In this paper, the single-precision floating-point multiplier is actually optimized by the booth-4 encoding for the trailing part (i.e., the 24-bit fixed-point multiplier). In addition, this paper also deals with the symbolic bit expansion of the booth-4 encoding. Since this 24-bit fixed-point multiplier is treated as a symbolic number by default, a simple processing should be done. af is processed as aff:{1′b0, af}. In this paper, bf is treated as the transcoded original code of booth-4 in the code as bf_b:{2′b00, bf, 1′b0} form, and then the transcoding process is performed corresponding to Table 1, hosting the symbols of each part (neg) and generating the transcoding code (zero, one, two). According to the transcode, the aff is operated accordingly, with zero being taken, one being unchanged, and two being shifted left by one. Then, determine whether the operation of taking the inverse plus one is needed according to the neg symbol. There is an important logic here such that the neg symbol is 0 by default under the premise of determining zero. This is an important logic point in the subsequent symbolic bit expansion [11].

In the case that the basic encoding has been completed, it is necessary to do another simplification of booth-4, which is used as a prediction of the booth algorithm with a rounding, again compressing its partial product [12]. Then, according to the partial product logical association of each line to do symbolic bit expansion simplification, here note that if there are zero cases, the front added symbolic bit neg default is 0, ∼neg is 1. So far, we get 13 partial product prod, the end of the first flow level, into the second level of flow.  Figure 5 shows the comparison of the partial product after the expansion with symbolic bits after the booth processing.

In the second level of flow, what this paper has to do is based on the first level of the partial product of 13 prods' multiple coverage compression to the last only one layer of product situation. According to the 3-2 compressor theory (2-2 compression is 3-2 compression in one additive to zero states), make add compression module; in the second level of flow in six levels cover the compression of 13 layers of prod so as to get the final result product. Therefore, a compression module needs to be added at each level to avoid bias. In the last level of the six-level overlay compression, the last two levels are added directly to obtain the final fixed-point 24-bit multiplication product using the system's built-in overfeed adder [13].  Figure 6 shows the compression coverage of the six-level level.

In the Wallace tree above, we have obtained the product of fixed-point multiplication results for the trailing part so that the symbolic bits, the order part, and the trailing part of the resultant floating-point number have been obtained. Nowadays, rounding and direct rounding are popular in precision, and the former scheme is adopted in this design. In the end, the first result of the final fixed-point product is judged to be 1 to determine the overflow of the ordinal code. If the first place of fixed-point product is 0, the order code exceeds 382 as the maximum overflow and is below 127 as the minimum overflow, and the fixed-point product result cf2<=[45:23] is extracted in the nonoverflow case. If the first place of the fixed-point product is 1, the order code beyond 381 is the maximum overflow, below 126 is the minimum overflow, and the result of extracting the fixed-point product in the nonoverflow case is cf5<=[46:24]. Then, do the precision constraint part, judge the latter bit of the extracted result part, and judge whether it is required as a feed. Here, it should be noted that the condition needs to be attached whether the extracted part is all one, or the order code is the maximum number 255, that is, whether the overflow result may be caused in the rounding state, if not, then the extracted part cf5 + 1. So, this paper gets a single-precision floating-point multiplier with the accuracy to meet the usage requirements. Complete the design requirements.

## 3. Results and Discussion

### 3.1. Code Logic Functional Verification

#### 3.1.1. Testbench Environment Creation

Here, in this paper, we first write the most basic single-precision floating-point multiplier, whose core 24-bit fixed-point multiplier uses the simplest shift-hosted binary multiplication, and here we can get a series of codes for single-precision floating-point multiplier. After writing the codes, we make the corresponding comparisons on the flowing water, citing the nonflowing water format and the flowing water format. And the source code is verified by the relevant logic, and the corresponding verification code is written in testbench, and the comparison output true for the code output is consistent with the MATLAB gold model production product result. See waveform in Figure 7 and logic verification in Figure 8.

As you can see, after the source code is written, the logic function is verified to be error free, and the accuracy is fully up to the requirements. The comparison between the waveform graphs of nonflowing and flowing formats also shows that the throughput in the flowing format is much larger than that in the nonflowing format so that the basic code is established, and the following is the code modification of the source code, adding the booth and Wallace tree modules, after which the combination and generation of partial product modules are optimized accordingly to achieve the desired goal.

#### 3.1.2. Logic Validation after Adding the Boothwallace Tree Module

In this paper, we add the optimized boothwallace module here to generate the final code, and then add and reduce the state of the running module, and use the original testbed environment to functionally verify the final code, and again compare the raw product of the code with the raw product in the MATLAB gold model database for numerical comparison. Figures 9 and 10 show the waveforms obtained from the verification.

Here, the verification related to the logic function of the code has been concluded in this paper, and the algorithm is extracted and analyzed for each parameter to verify whether it achieves the expected effect of this paper when the use of the function can be confirmed without errors.

### 3.2. Comparison of Power Consumption of Fixed-Point Multipliers

Here, in this paper, we first analyze the power consumption of the fixed-point multiplier in this paper and take out the 24-bit fixed-point multiplier of the most basic fmpy shift-hosting direct sum, the multiplier of the simple added booth module and Wallace module, and finally, the 24-bit fixed-point multiplier of boothwallace after optimization in this paper. Because these are all combined logic parts, this paper sets its max_delay to 0.5 ps, that is, according to the frequency of 2 GHz work, combines logic area, and measures its power consumption data. The data are recorded and compared at 25c, 85c, and 125c for three temperature process angles to get a relatively detailed report. They are displayed as Tables 2, 3, and 4, respectively.

The obtained statements are organized to obtain area (Figure 11) and power consumption comparison (Figure 12) for the three fixed-point module algorithms corresponding to different temperature process angles.

Here, we get the corresponding power consumption data of each fixed-point multiplier module. This paper can analyze that, with the maximum delay parameter set, the area of the combinational logic part of the original fmpy_24 fixed-point multiplier is the smallest under the process angle model of each temperature, resulting in its power consumption in all aspects being lower than the normal value. The area of the fmpy_24 fixed-point multiplier is the smallest, resulting in a lower than normal power consumption in all aspects. The area of the fmpy_24 fixed-point multiplier is increased by simply adding the booth code and the Wallace tree module, and the power consumption is increased accordingly. Since the fixed-point multiplication part is the core operation module of single-precision floating-point multiplication, the optimized power consumption and area of the fixed-point multiplication module are of great significance for the power consumption and area of the entire single-precision floating-point part. The following is a comparison of the power consumption of the single-precision floating-point section.

### 3.3. Single-Precision Floating-Point Multiplier Power Consumption Comparison

After the analysis of each bit of data of the internal module 24-bit fixed-point multiplier module was carried out above, here the analysis of power consumption data is done for the source code fmpy, the algorithm of adding booth and Wallace normally, and the final algorithm of the optimized boothwallace module to get the final power consumption statement. The different temperature process angles from 25c, 85c to 125c are shown in Tables 5–7. In addition to the data on the above aspects, this paper adds a record on the peak power, which helps to clarify the choice of chip power. In the integrated netlist section of this paper, the timing.sdc file is designed with an excitation of 0.5 ps, reaching the final measurement frequency of 2 GHz.

The combined and noncombined area comparison of the floating-point multiplier for the three algorithms is obtained in Figure 13, the total power consumption comparison in Figure 14, and the peak power comparison in Figure 15.

From the above tables, we can see that after the modification of the algorithm in the noncombination of the area is greatly reduced, although the combination of logic part compared to the most just fmpy algorithm way to increase, but adding combinatorial logic modules to the fixed-point modules will definitely create excess losses. The area of the floating-point algorithm is still much smaller than that of the fmpy algorithm of the shift-hosting method and the normal algorithm of simply adding the booth and Wallace modules. The total power of the modular algorithm of simply adding booth and Wallace is much lower than the original shift-hosting fmpy algorithm in the power analysis, with a reduction of 45.95%, while the optimized boothwallace algorithm module total power algorithm compared to the shift-hosting fmpy algorithm reduction of 58.69%, proving that optimizing Wallace will get very significant power savings, and on top of that adding a symbolic bit expansion module there is a not insignificant secondary improvement. In the peak power measurement, in various temperature process angles, the peak power reduction of the normal algorithm with the simple addition of the booth and Wallace modules and the optimized boothwallace algorithm compared to the original shifted hosting fmpy algorithm are 3.79% and 7.97%, respectively, showing that the optimized algorithm also has a very significant improvement in peak power, which can make it a more generous choice in terms of power supply. At this point, the design fully meets the usage requirements.

The final result comes down to the resulting integrated netlist picture and cell diagram in Figure 16.

## 4. Conclusion

At this point in the paper, the single-precision floating-point multiplication algorithm has been logically designed and ultimately power-optimized through a series of rigorous verification and simulation processes. From source code writing, modification, verification on various platforms, synthesis, simulation, to the final experimental data, a comparative analysis of the experimental and control groups on multiple databases is performed. By using the symbolic bit expansion method to predict the partial product caused by the booth-4 code by rounding, the area of the resulting partial product tree is reduced. Then, the corresponding add operation and storage area are reduced in the covering structure of the Wallace tree, achieving the requirement of reducing the area and reducing power consumption. At this point, the algorithm design meets the expected requirements.

## Figures and Tables

**Figure 1:** Intel's microprocessor core-level.

**Figure 2:** Conventional multiplier design.

**Figure 3:** Design verification and simulation flow.

**Figure 4:** Single-precision floating-point multiplication structure.

**Figure 5:** Schematic diagram of symbol bit expansion.

**Figure 6:** (a) The first-level compression diagram. (b) The second-level compression diagram. (c) The third-level compression diagram. (d) The fourth-level compression diagram. (e) The fifth-level compression diagram. (f) The sixth-level direct overfeed summation.

**Figure 7:** Logic output diagram of flowing and nonflowing water.

**Figure 8:** Logic function verification diagram.

**Figure 9:** Optimized logic output diagram for flowing and nonflowing water.

**Figure 10:** Final code logic verification diagram.

**Figure 11:** Comparison of the combined area of fixed-point modules.

**Figure 12:** Comparison of total power consumption of fixed-point modules at three temperature process angles.

**Figure 13:** Area of combined and noncombined floating-point multiplier modules.

**Figure 14:** Comparison of total power consumption of floating-point multipliers at three temperature process angles.

**Figure 15:** Comparison of floating-point multiplier spike power consumption at three temperature process angles.

**Figure 16:** Integrated results' netlist diagram.

**Table 1:** Booth-4 transcoding table.

*X*_2*i*+1_ *X*_2*i*_ *X*_2*i*−1_	Part of the product *PP*_[*n* − 1 : 1]_	NEG	Z	*B*_1_	*B*_2_
000	+0 *∗* Y	0	1	1	0
001	+1 *∗* Y	0	1	0	1
010	+1 *∗* Y	0	0	0	1
011	+2 *∗* Y	0	0	1	0
100	−2 *∗* Y	1	0	1	0
101	−1 *∗* Y	1	0	0	1
110	−1 *∗* Y	1	1	0	1
111	−0 *∗* Y	1	1	1	0

**Table 2:** Power consumption table of each fixed-point multiplier of 25c.

2 GHz (TC-25C)	max_delay	Area (combination)	Power
fmpy_24	0.5	298.752	4.159*E* − 06
normal_24	0.5	529.4208	2.934*E* − 04
boothwallace_24	0.5	324.2592	1.923*E* − 04

**Table 3:** Power consumption table of each fixed-point multiplier of 85c.

2 GHz (TCH-85C)	max_delay	Area (combination)	Power
fmpy_24	0.5	298.752	2.894*E* − 05
normal_24	0.5	529.4208	2.947*E* − 04
boothwallace_24	0.5	324.2592	2.116*E* − 04

**Table 4:** Power consumption of each fixed-point multiplier of 125c.

2 GHz (WC-125C)	max_delay	Area (combination)	Power
fmpy_24	0.5	298.752	2.345*E* − 05
normal_24	0.5	529.4208	3.397*E* − 04
boothwallace_24	0.5	324.2592	2.309*E* − 04

**Table 5:** 25c single-precision floating-point multiplier power consumption table.

2 GHz (TC-25C)	Area (nonportfolio)	Area (combination)	Total power	Peak power
fmpy	568.5504	375.9168	3.016*E* − 04	0.1556
Naomal	71.1552	560.0448	1.630*E* − 04	0.1493
boothwallace	67.1443	290.8974	1.246*E* − 04	0.1432

**Table 6:** 85c single-precision floating-point multiplier power consumption table.

2 GHz (TC-25C)	Area (nonportfolio)	Area (combination)	Total power	Peak power
fmpy	568.5504	375.9168	3.780*E* − 04	0.1586
Naomal	71.1552	560.0448	2.133*E* − 04	0.1496
boothwallace	67.1443	290.8974	1.562*E* − 04	0.1439

**Table 7:** 125c single-precision floating-point multiplier power consumption table.

2 GHz (TC-25C)	Area (nonportfolio)	Area (combination)	Total power	Peak power
fmpy	568.5504	375.9168	3.192*E* − 04	0.1136
Naomal	71.1552	560.0448	1.894*E* − 04	0.1025
boothwallace	67.1443	290.8974	1.396*E* − 04	0.1012

## Data Availability

All data included in this study are available upon request to the corresponding author.
